# The role of macrophages in polycystic ovary syndrome: A review

**DOI:** 10.1097/MD.0000000000042228

**Published:** 2025-04-25

**Authors:** Li Li, Yubo Xiao, Wenwei Wen, Qi Liu, Le Wei, Pinyue Liu, Ming Li

**Affiliations:** a Department of Histology and Embryology, Hunan University of Medicine, Huaihua, China; b School of Public Health and Laboratory Medicine, Hunan University of Medicine, Huaihua, China; c Department of Orthopedics, Sanming First Hospital Affiliated to Fujian Medical University, Sanming, Fujian, China.

**Keywords:** insulin resistance, macrophage, MIF, PCOS, PCOS endocrine feature

## Abstract

Polycystic ovary syndrome (PCOS) is a common endocrine disorder among fertile women, which is influenced by genetics and environment. A recent study revealed that PCOS patients were in a chronic inflammatory state, and they had abnormally activated macrophages. This paper introduces the relationship between PCOS and macrophages. The forkhead box protein O1 (FOXO-1), migration inhibitory factor, sympathetic conservation disorder, and vitamin D are believed to influence macrophages in PCOS. There is evidence that PCOS-associated abnormalities are associated with macrophages, including insulin resistance, obesity, hyperandrogenism (HA), hyperhomocysteinemia (HHcy), cardiometabolic disorder and gut microbiota dysbiosis. This review summarizes the research status of macrophages in PCOS. Macrophages might be a potential PCOS treatment candidate.

## 1. Introduction

Polycystic ovarian syndrome (PCOS) is a multi-system disorder, it has complex reproductive, metabolic, and psychological characteristics.^[1]^ Since this syndrome can lead to infertility, insulin resistance (IR), obesity, cardiovascular diseases, and other endocrine disorders, it is no longer simply considered an ovarian disease.^[2]^ Immune dysfunction has been summarized as a key factor in PCOS occurrence and development.^[3]^ There is local ovarian inflammation in patients with PCOS, which is detrimental to the development of follicles.^[4]^ In the ovary of PCOS, inflammation-related cytokines interact.^[5]^ PCOS is related to an increase in interleukin-18 (IL-18), monocyte chemoattractant protein-1 (MCP-1) and macrophage inflammatory protein 1α (MIP-1α).^[6]^ Immunoinfiltration analysis of collected PCOS samples showed a strong positive correlation between activated natural killer cells (NK) and memory B cells, with the strongest negative correlation between neutrophils and monocytes. The RT-qPCR results showed overexpression of CD163, TREM1, and TREM2 genes.^[7]^ A large clinical study by Liu et al showed that overweight PCOS patients had higher CD68^+^ and CD163^+^ macrophage levels in their endometrium than normal women.^[8]^ The number of immune cells in the endometrium of women with PCOS increased, resulting in a low-grade chronic inflammation condition.

Inactivated macrophage is M0 type. The phenotypes of activated macrophages are M1 macrophages and M2 macrophages (Fig. 1). M1 macrophages start and sustain inflammatory responses during the maintenance of body homeostasis, and an excessive immune response can result in chronic inflammation. M1 macrophages are activated by lipopolysaccharide (LPS) and interferon (IFN)-γ, and induce activation and secrete pro-inflammatory cytokines: tumor necrosis factor (TNF)-α, IL-1, IL-6, inducible nitric oxide synthase (iNOS).^[9]^ The M2 macrophages are involved in tissue repair and immune tolerance. M2 macrophages are induced by cytokines such as IL-4 and IL-13 through activation of signal transduction and activator of transcription 6.^[10]^ M2 macrophages secrete IL-10, arginase and transforming growth factor-β to inhibit inflammatory reactions.^[11]^ M2 macrophage is also an effective phagocyte. The purpose of M2 macrophage is to eliminate debris and induce wound healing and angiogenesis.

**Figure 1.** M0 macrophages were polarized towards M1 and M2 respectively under different stimuli. M0 macrophages were polarized towards M1 induced by LPS and IFN-γ, and activated M1 macrophages could release TNF-α, IL-1, IL-6 and iNOS, which involved in proinflammation and tissue injure. M2 macrophages induced and activated by IL-4 and IL-13 through activation of STAT6 then secreted IL-10 and TGF-β, which involved in inflammation and tissue repair. IFN-γ = interferon-γ, IL = interleukin, iNOS = inducible nitric oxide synthase, STAT = signal transduction and activator of transcription, TNF = tumor necrosis factor.

Macrophages participate in PCOS chronic inflammatory infiltration. A study by Xie et al found that the number of peripheral and splenic neutrophils and M1 macrophages was higher in PCOS mice.^[12]^ A study by Wang et al demonstrated that M1 macrophages in the ovary of PCOS mice were significantly increased, which was accompanied by a systemic inflammatory response and an abnormal ovulation cycle.^[13]^ These results indicated that there was an imbalance between activated M1 and M2 macrophages in PCOS. In the presence of a local cytokine environment, both M1 and M2 macrophages can undergo reversible functional changes.^[14]^ Macrophages are believed to play a central role in PCOS pathogenesis. One of the most researched mechanisms is diet-induced alterations in the microbiome (dysbiosis) that cause release of LPS and increased gastrointestinal barrier permeability. LPS binds with LPS binding protein which activates toll-like receptor (TLR)-4 on submucosal macrophages.^[5,15]^ This activates NF-κB and results in the release of inflammatory cytokines in different tissues throughout the body. Therefore, it is important to regulate the proportion of macrophages M1 and M2 in patients with PCOS. The purpose of this article is to discuss the relationship between macrophages and PCOS from 2 perspectives: the key factors affecting macrophages in PCOS (Fig. 2), and the endocrine characteristics that may be associated with macrophages in PCOS (Fig. 3).

**Figure 2.** M1 macrophages aggregation in PCOS ovary. The increase of FOXO-1 and MIF, the decrease of VD and sympathetic innervation disorder promoted the M1 macrophages aggregation in PCOS ovary. FOXO-1 = forkhead box protein O1, MIF = migration inhibitory factor, PCOS = PCOS = polycystic ovary syndrome, VD = Vitamin D.

**Figure 3.** Mechanism network of macrophage regulation of PCOS complications. HHcy accelerated cardiovascular disease, such atherosclerosis by promoting lipid accumulation and mediating cholesterol efflux of macrophage. HHcy lead to the imbalance of M1/M2 macrophages by inhibiting intermedin expression, which promoted IR and obesity. Monocyte-derived and polarized M1 macrophages were production of TNF-α and IL-6. Increased TNF-α and IL-6 promoted IR and atherosclerosis.In addition to IR and obesity, and increased morbidity of cardiovascular disease, hyperandrogenism could also lead to gut microbiota dysbiosis, which impaired glucose metabolism and eventually caused IR. HHcy = hyperhomocysteinemia, IR = insulin resistance, PCOS = polycystic ovary syndrome, TNF = tumor necrosis factor.

## 2. The key factors affecting macrophages in PCOS

### 2.1. FOXO-1

The transcription factor FOXO-1 is critical for regulating cytokine and chemokine secretion.^[16]^ FOXO-1 protein can be phosphorylated by the c-Jun N-terminal kinase (JNK) or macrophage-stimulated protein-1, which results in FOXO-1 protein entering the nucleus, blocking the effect of phosphoinositol 3-kinase/protein kinase B (PI3K/PKB).^[17]^ It has been shown that FOXO-1 was overexpressed in macrophages, which were infected with parasites in the host cell.^[18]^ Besides increasing cell apoptosis, FOXO-1 also promotes TLR-4, noncanonical nuclear factor (NF)-κB and IL-1β and decreases IL-10 secretion. FOXO-1 activates the maintenance of homeostasis, and regulates neutrophils, macrophages and pro-inflammatory signaling molecules in mucosal tissues.^[19]^ Li research showed that high levels of FOXO-1 phosphorylation were related to the generation of IL-6, IL-1β, and TNF-α in macrophages of PCOS patients. FOXO-1 phosphorylation enhanced TLR-4 signaling in response to LPS, while knockdown of FOXO-1 reduced insulin-induced glucose uptake in PCOS macrophages.^[20]^ Pro-inflammatory responses are primarily triggered by glucose-mediated oxidative stress.^[21]^

### 2.2. Migration inhibitory factor

Macrophage migration inhibitory factor (MIF) is a multifunctional cytokine that activates macrophages and T cells.^[22]^ MIF regulates glucocorticoids-induced annexin 1 expression and arachidonic acid release from macrophages.^[23]^ MIF binds to the receptors CD74/CD44 and CXCR2, 4 and 7 in an autocrine and paracrine manner. A pro-inflammatory response is also mediated by MIF through downstream activation of extracellular signal-regulated kinase (ERK) 1, 2, AMPK, and AKT.^[24]^ More and more evidence showed that there was a link between MIF and PCOS. Researchers reported that increased MIF activated the NF-κB pathway in the ovary, which led to the elevation of inflammation and related inflammatory markers.^[25]^ PCOS women have significantly higher plasma MIF levels than normal women. There was a positive correlation between MIF and luteinizing hormone, free testosterone, body mass index (BMI), high-sensitivity C-reactive protein (hs-CRP), and IR homeostasis model assessment in PCOS women.^[26]^ There was a significant difference in plasma MIF levels between obese and nonobese women with and without PCOS, and MIF expression was significantly increased in obese PCOS women.^[27]^ Khashchenko research also revealed that the MIF of overweight PCOS adolescents was significantly higher than that of normal girls.^[28]^ These results indicated that macrophages were involved in chronic inflammatory infiltration due to the increase in visceral fat. Zhou et al found that MIF participated in the pathogenesis of PCOS via the mitogen-activated protein kinase signaling pathway.^[29]^

### 2.3. Sympathetic innervation disorder

An important function of the sympathetic nervous system is to innervate the ovary. Sympathetic nerve fibers were found to regulate androgen secretion and follicle maturation in the ovary in an animal study.^[30]^ Corticotrophin-releasing hormone (CRH) and nerve growth factor (NGF) are the modulators for the actions of the sympathetic nervous and immune systems. CRH, NGF, and IL-17α in serum of patients with PCOS were significantly lower than in the control group.^[31]^ IL-1α and IL-1β significantly increased in the PCOS group. Modulation of the immune-endocrine function by the peripheral sympathetic nervous system might have implications for understanding the pathophysiology of PCOS. Figueroa et al used culture media of macrophages from PCOS rats and PCOS rats with superior ovarian nerve (SON) section (PCO-SON rats) were used to stimulate in vitro intact ovaries.^[32]^ Their results showed that compared with PCOS rats, PCO-SON rats’ macrophages released less TNF-α and nitric oxide. Furthermore, SON partially reduced the expression of kisspeptin and NGF in PCOS rats. SON is involved in the second modification of immune and neurotransmitter systems, as well as influencing the production of ovarian steroids. However, Linares R demonstrated that unilateral sectioning of the SON could restore ovulation of the innervated ovary.^[33]^ Therefore, SON disorder will seriously affect the secretion of inflammatory factors and hormones of macrophages in PCOS.

### 2.4. Vitamin D

Vitamin D (VD) has become a key regulator of the innate immune response. CYP27B1 (cytochrome enzymes) expression in macrophages was induced by immune-specific input, resulting in the local production of 1,25-dihydroxyvitamin D at the infected site.^[34]^ PCOS women generally lack VD. There is a negative correlation between serum VD levels and PCOS metabolism and hormonal disorders. PCOS women receiving VD treatment had increased endometrial thickness and increased pregnancy rates.^[35]^ Low levels of VD have been associated with an increased risk of IR and diabetes in PCOS patients.^[36]^ In the experiment of Maktabi et al, 12 weeks VD supplementation significantly reduced fasting blood sugar, insulin and increased quantitative insulin sensitivity.^[37]^ Trummer C, however, found that VD supplementation had no significant effect on metabolic and endocrine parameters, such as the area under the plasma glucose curve in patients with PCOS.^[38]^ Various immune cells, including lymphocytes, monocytes, macrophages, and dendritic cells, express VDR and VD metabolic enzymes.^[39]^ The activated macrophages and monocytes strongly express CYP27B1, which converts 25(OH)D into 1,25(OH)_2_D.^[40]^ The production of 1,25(OH)_2_D by macrophages could up-regulate the expression of cathelicin LL-37, which affected the function of nearby lymphocytes.^[41]^ The effect of macrophages derived cytokines on PCOS were conducted during the COVID-19 pandemic. PCOS patients increased the expressions of the basic macrophage activation markers CXCL5, CD163 and MMP-9, while the protective macrophage marker CD200 decreased. Their study discovered that VD-deficient PCOS patients had higher basal macrophage activation, which was associated with decreased CD80 and IFN-γ.^[42]^

## 3. Macrophage in PCOS on endocrine feature

### 3.1. Insulin resistance and obesity

Insulin resistance is defined as a diminished biological response to circulating insulin.^[43]^ Regardless of age, the prevalence of gestational diabetes, impaired glucose tolerance and type 2 diabetes are significantly increased in PCOS, with risk independent of, yet exacerbated by, obesity.^[44,45]^ About 75% of PCOS patients have impaired insulin action.^[46]^ Those with PCOS who are overweight are more likely to require regular monitoring and analysis of their blood glucose levels.^[47]^ In a clinical study by Khashchenko, normal weight PCOS girls with IR had lower levels of C-reactive protein, leptin, and malondialdehyde and higher levels of soluble Fas ligand (sFasL) compared to healthy girls in the control group. IR in obese PCOS girls was associated with higher levels of IL-18, activated oxidative stress, as well as systemic inflammation.^[28]^ Studies have shown a connection between IR, obesity, and macrophages. Obesity’s pro-inflammatory state promotes IR and atherosclerosis. Glucose could trigger oxidative stress and the monocyte (MNC) inflammatory response in PCOS women. Hypoxia-related adipocyte death caused by adipose tissue expansion promotes MNC influx into the stromal vascular compartment. These MNCs undergo morphological changes and become resident macrophages.^[48]^ MNC derived macrophages are the main production source of TNF-α and IL-6 in adipose tissue. TNF-α is a known IR mediator, and IL-6 is obviously involved in atherosclerosis promotion.^[49]^ Su et al treated PCOS mice with testosterone to induce IR. IR activated NF-κB, promoted the expression of IL-6 and MCP-1, and transformed macrophages to the M1.^[50]^ Visfatin is an adipokine, it exerts an insulin-like effect by binding to the insulin receptor-1 and has a hypoglycemic effect.^[51]^ There was no significant increase in plasma visfatin levels or visfatin gene expression in monocytes and monocyte-derived macrophages in peripheral blood of PCOS patients in Zhang experiment.^[52]^ Considering their findings, studies of the effects of macrophages on PCOS or IR should examine macrophages in tissues rather than peripheral blood. The study by Liu examined the immune cells in the endometrium of PCOS women with IR, determining that CD56^+^ NK cells and CD163^+^ M2 macrophages were positively correlated with the quantitative insulin sensitivity index (QUICKI), indicating that there was an association between immune cells in the endometrium and IR.^[5]^ Betatrophin therapy experiments in vitro and in vivo demonstrated that hepatocytes and macrophages interacted with cellular to regulate dystrophin levels in PCOS women with IR.^[53]^

### 3.2. Hyperandrogenism

Hyperandrogenism (HA) is one of the most prominent endocrine features of PCOS. Its clinical manifestations include obesity, acne, hirsutism, and androgenetic alopecia. Official organizations divide PCOS into 4 types according to HA. The risk of cardiovascular disease in PCOS is more closely associated with the HA phenotype.^[54]^ There is an abnormal steroid secretion defect in most PCOS patients with HA, resulting in abnormal folliculogenesis and a failure of dominant follicle selection.^[55]^ In addition to affecting granulosa cell function and follicle development, excessive androgens cause obesity and IR, inducing a vicious cycle of PCOS development.^[56]^ Studies have found that HA may be related to immunity. In HA PCOS granulosa cell samples, Gao et al identified 271 differentially expressed genes enriched in immune activation and inflammatory response.^[57]^ PCOS patients are commonly obese, and HA can stimulate the expression of pro-inflammatory mediators in adipocytes. Su demonstrated that testosterone activated IL-6 and MCP-1 by phosphorylating ERK1/2 and NF-κB.^[58]^ Researchers have found an association between HA and macrophages in PCOS patients. The research of Li et al showed that testosterone increased kisspeptin expression. Pro-inflammatory cytokines and nitrite released in excess of androgen stimulated macrophages, further impairing their vitality and increasing apoptosis.^[59]^ However, the study did not specify whether it inhibited M1 or M2 macrophage apoptosis. Lima PDA research demonstrated that HA increased ovarian chemerin, 5α-dihydrotestosterone (DHT) altered follicle dynamics while increased the M1: M2 macrophages ratio in antral and preovulatory follicles. While ovarian M1 macrophages expressing chemokine-like receptor 1 (CMKLR1) were increased, CMKLR1^+^ monocytes, which migrated toward chemerin-rich environment, were markedly decreased after 15 days of DHT, induced granulosa cell apoptosis.^[60]^ Chen et al research suggested that the high androgen microenvironment could promote the activation of M1 by ovarian macrophages, which may be related to the reprogramming of macrophage glucose metabolism. The increased secretion of pro-inflammatory cytokines by macrophages in the high androgen microenvironment can impair the normal function of granulosa cells and interfere with normal follicular growth and development.^[61]^ Higher frequency of NK cells and higher levels of IFN-γ and TNF-α were observed in the uterus of androgen exposed mice, while NK cells in visceral adipose tissue and spleen showed higher levels of CD69 expression, and the mice exhibited IR.^[62]^

### 3.3. Hyperhomocysteinemia

Homocysteine (Hcy) is an amino acid that requires vitamin B12 and folic acid for its metabolism. Vitamin B12 and folic acid deficiency cause hyperhomocysteinemia (HHcy).^[63]^ The coexistence of HA and HHcy in PCOS patients can lead to atherosclerosis.^[64]^ According to Chakraborty research, HHcy could cause miscarriage in women with PCOS. With PCOS and HHcy, 4.49% of women had cardiovascular disease 3 years after delivery.^[65]^ Studies have shown that HHcy was related to macrophages in PCOS. Proprotein convertase subtilisin kexin 9 promoted lipid accumulation by inhibiting ATP binding cassette transporter A1 and G1 (ABCA1 and ABCG1), mediated cholesterol efflux from macrophages and accelerated atherosclerosis with HHcy.^[66]^ HHcy also stimulated an increase in M1/M2 macrophage ratio, leading to more inflammatory features. In contrast, regular exercise reduces the M1/M2 ratio, reducing the inflammatory phenotype.^[67]^ A study conducted by Qi demonstrated that HHcy inhibited estrogen’s ability to regulate the polarization pathway of macrophages in PCOS mice by further enhancing the IR.^[68]^ The calcitonin family peptide intermedin (IMD) was also reported to be lower in plasma and adipose tissue of mice with HHcy. IMD reversed the elevated Hcy ratio in M1/M2 macrophages by inhibiting AMP-activated protein kinase activity, which resulted in reduced endoplasmic reticulum stress and a reduction in inflammatory responses, and improved IR in mice with HHcy.^[69]^

### 3.4. Cardiometabolic disorder

There is an increased risk of PCOS patients developing coronary artery disease, atherosclerosis, and other cardiometabolic diseases.^[70]^ PCOS patients often have elevated levels of total cholesterol and high-density lipoprotein cholesterol (HDL-C). Roe A revealed that women with PCOS had a significantly higher BMI and blood pressure, as well as a 7% lower normalized cholesterol efflux capacity.^[71]^ Her study demonstrated that PCOS was also associated with atherosclerosis, including increased quantities of large very-low-density lipoprotein particles, very-low-density lipoprotein, and small low-density lipoprotein cholesterol particles.

A regular menstrual cycle causes macrophage activation to fluctuate regularly. However, in PCOS patients, this dynamic pattern is attenuated, leading to chronically activated macrophages in the ovaries. PCOS is associated with vascular inflammation and atherosclerosis because of proinflammatory activation and dysregulated cholesterol metabolism in the monocyte-macrophage system.^[72]^ In PCOS patients, macrophages are attenuated in response to multiple hormonal stimuli, and HDL cholesterol efflux capacity is significantly reduced.^[73]^ A study conducted by Dokras A found that women with PCOS reduced cholesterol efflux capacity, resulting in a decrease in HDL-C cholesterol levels, which were not conducive to cholesterol excretion.^[74]^ Chronically activated macrophages together with impaired serum high-density lipoprotein cholesterol function accelerate PCOS-related cardiometabolic risk. PCOS could affect cardiovascular health in women by promoting myocardial macrophage accumulation and post-MI cardiac remodeling.^[75]^ Single gene analysis suggested that the matrix metallopeptidase 9 (MMP-9) and P2RY13 might be involved in metabolism and inflammation responses. Zhang et al identified MMP-9 and P2RY13 as the biomarkers and developed a new nomogram for early diagnosing cardiometabolic disorder based on them in PCOS patients.^[76]^

### 3.5. Gut microbiota dysbiosis

The gut microbiota affects numerous organs and pathways outside the gastrointestinal tract. Microbiota play a significant role in the female reproductive endocrine system via their interactions with estrogen, androgen, insulin, and other hormones.^[77]^ The excessive levels of testosterone caused by HA may affect the composition of the gut microbiota of women suffering from PCOS. Based on regression analysis, PCOS mice with decreased abundance of several genera showed increased circulating testosterone levels and impaired glucose metabolism.^[78]^ According to Qi et al, PCOS patients had a significantly increased level of Bacteroides vulgaris on their gut microbiota, which was accompanied by a significant decrease in glycodeoxycholic acid and taurine ursodeoxycholic acid. Fecal microbiota transplanted into recipient mice from women with PCOS caused increased ovarian dysfunction, IR, a decrease in IL-22 secretion, and infertility.^[79]^ After supplementing with IL-22, PCOS mice improved the above characteristics. Diet is a major regulator of the intestinal microbiota. Rodriguez Paris V et al found that various diets that contain protein, carbohydrates and fat significantly improved the α and β diversity and ratio of Bacteroides acidifaciens in PCOS mice.^[80]^ In their study, they found that transplanting gut microbiota from normal mice to PCOS mice enhanced the gut microbiota structure and decreased body fat content. However, it did not significantly alleviate PCOS symptoms. According to them, it may be because each PCOS mouse model has its own gut microbiota. A single type of flora transplantation will not meet the needs of every mouse model. Huang et al observed that in PCOS mice, intestinal Achmania decreased, Gram-negative bacteria (Desulfovibrio and Burkholderia) increased, and serum LPS and IFN-γ increased.^[81]^ LPS and IFN-γ could induce macrophage pyroptosis in the mouse ovary. Macrophage pyroptosis destroyed estrogen production and promoted granulosa cell apoptosis. By knocking down Gasdermin D and inhibiting macrophage pyroptosis, PCOS can be significantly improved. They also found that Metformin could increase the abundance of Akkermansia in the intestinal tract and reduce the serum IFN-γ, inhibit the scorch of ovarian macrophages, thereby improving PCOS. HeQi San (HQS) could mediate the abundance of gut microbiota in mice with PCOS. Besides, HQS had the effect of anti-inflammation and inhibited macrophage M1 polarization.^[82]^

## 4. Conclusion

PCOS is a common neuroendocrine, reproductive, and metabolic disorder. Studies showed that PCOS patients were chronically affected by inflammation. This review found evidence for macrophage role in PCOS pathogenesis and pathophysiology. FOXO-1, MIF, synaptic activation, and VD have been shown to be involved in macrophage dysregulation in PCOS. Macrophages regulate several PCOS endocrine complications, including IR, obesity, HA, HHcy, gut microbiota dysbiosis and cardiovascular disease. These endocrine complications are interconnected. Future research should investigate therapeutic options of PCOS that target these mechanisms to reduce macrophage activation and inflammation.

## Acknowledgments

We thank all the listed authors in the manuscript.

## Author contributions

**Conceptualization:** Pinyue Liu.

**Data curation:** Yubo Xiao, Le Wei.

**Formal analysis:** Yubo Xiao.

**Methodology:** Li Li, Qi Liu.

**Writing – original draft:** Qi Liu, Pinyue Liu.

**Writing – review & editing:** Yubo Xiao, Wenwei Wen, Ming Li.
